This article has been retracted.

# Phytochemical screening, HPLC fingerprinting and *in vitro* assessment of therapeutic potentials of different apricot cultivars against diabetes, Alzheimer's disease and cancer

**DOI:** 10.1016/j.heliyon.2024.e38673

**Published:** 2024-09-28

**Authors:** Zahid Nabi Sheikh, Vikas Sharma, Shilpa Raina, Prashant Bakshi, Rizwan yousuf, Ali Zari, Talal A. Zari, Khalid Rehman Hakeem

**Affiliations:** a Division of Fruit Sciences, Sher-e-Kashmir University of Agricultural Sciences and Technology, Jammu, 180009, J&K, India; b Division of Biochemistry, Sher-e-Kashmir University of Agricultural Sciences and Technology, Jammu, 180009, J&K, India; c School of Applied Sciences, Shri Venkateshwara University, Gajraula, UP, India; d Division of Statistics and Computer Sciences, Sher-e-Kashmir University of Agricultural Sciences and Technology, Jammu, 180009, J&K, India; e Department of Biological Sciences, Faculty of Science, King Abdulaziz University, Jeddah, 21589, Saudi Arabia; f Princess Dr. NajlaBint Saud Al-Saud Center for Excellence Research in Biotechnology, King Abdulaziz University, Jeddah, 21589, Saudi Arabia; g Department of Public Health, Daffodil International University, Dhaka, 1341, Bangladesh; h University Centre for Research and Development (UCRD), Chandigarh University, Punjab, India

**Keywords:** Bioactive, Anti-diabetic, Anti-Alzheimer, Anti-Cancer, α-amylase, α-glucosidase, Acetylcholinesterase

## Abstract

Plant-based natural compounds are widely used to treat various ailments owing to their readily availability and minimal adverse effects. This study aimed to perform qualitative and quantitative biochemical profiling and assess the in vitro anti-diabetic, anti-Alzheimer, and anti-cancer activities of various apricot (*Prunus armeniaca*) cultivars. High-performance liquid chromatography (HPLC) was utilized to determine the concentrations of bioactive compounds across 10 distinct apricot cultivars. Initial phytochemical screening revealed a significant content of secondary metabolites. Subsequently, methanolic extracts from these cultivars were evaluated for their therapeutic potential against several human cancer cell lines, including prostate cancer (PC-3), lung cancer (A-549), breast cancer (MCF-7), cervical cancer (HELA), and kidney cancer (HEK). Notably, the breast cancer cell line MCF-7 showed a pronounced inhibition rate post-treatment with the apricot extracts. Correlation analysis exhibited phenols are highly correlated with flavonoids (r = 0.92), DPPH (r = 0.95), and alpha-amylase (%) inhibition (r = 0.96), and showed a significant correlation with other parameters. Principal Component Analysis (PCA) revealed that PC1 explained 43.31 % of the variance, while PC2 explained 12.88 %, together explaining 80.033 % of the total variance. PC1 was identified as the dominant axis, indicating the primary pattern of variation among the variables. Hierarchical Cluster Analysis (HCA) divided the cultivars into 2 main clusters, with cluster 2 further subdivided into various sub-clusters and sub-sub-clusters. This analysis highlighted distinct genetic similarities and differences among the apricot cultivars. Among the tested cultivars, ‘Irani’ and ‘Tilton’ were found to contain the highest levels of bioactive constituents. This research marks the first comprehensive examination of the impacts of these two apricot cultivars. The findings from this study provide a robust scientific foundation for the future isolation and purification of therapeutic compounds, potentially leading to their application in pharmaceuticals or dietary supplements. This research contributes significantly to the understanding of the pharmacological properties of apricot cultivars and establishes a basis for further investigation into their clinical benefits.

## Highlights

• This study introduces two less commonly studied apricot varieties, Irani and Tilton, and highlights their effective health benefits, particularly in anti-cancer properties against the breast cancer cell line (MCF-7).
• The research reveals substantial variability in phytochemical content among different apricot cultivars, emphasizing the importance of genetic factors and environmental conditions in determining bioactive compound concentrations.
• Irani and Tilton cultivars demonstrate significant inhibitory activity against diabetic enzymes and acetyl cholinesterase, suggesting potential therapeutic applications in managing diabetes and neurodegenerative diseases like Alzheimer's.
• The study underscores the presence of various bioactive constituents, including alkaloids, saponins, and tannins, in apricot extracts, which contribute to their health-promoting effects and offer promising alternatives for disease management.

## 1 Introduction

The global perspective on daily nutrition is undergoing significant transformation, with increasing emphasis on concepts such as “functional foods,” “superfoods,” and “novel foods.” There's also a focus on developing new additives and nutritional supplements derived from natural plant bioactive components [1,2]. A notable strategy gaining attention involves leveraging nature-derived remedies from medicinal plants [3]. Bioactive plant components are emerging as popular natural alternatives across various industries, including pharmaceuticals, cosmetics and food [4]. Their non-toxic nature, potential effectiveness and renowned antioxidant capabilities are instrumental in devising treatments for numerous diseases [5,6]. Exposure to free radicals, such as reactive oxygen and nitrogen species (ROS/RNS), triggers an oxidative burst, leading to harmful outcomes like lipid peroxidation, protein denaturation, reduced enzyme activity and cell shrinkage. These effects collectively contribute to the progress of severe conditions, including cancer, diabetes mellitus and neurodegenerative diseases. Such oxidative stress can be mitigated through endogenous or exogenous antioxidant mechanisms [[7], [8], [9]]. Additionally, the rise in antibiotic resistance has escalated the threat of new infectious and chronic diseases, causing numerous epidemics with devastating health impacts [10,11]. Medicinal herbs and plants are increasingly recognized for their potential benefits, high safety profile, minimal side effects and the growing consumer interest in natural compounds for disease treatment [12]. The bioactive molecules in these botanicals are known to modulate signaling pathways associated with acute or chronic inflammation [13]. This burgeoning interest in identifying novel plant-based components for their bioactive properties has highlighted fruits like the *Prunus armeniaca* (apricot) for its traditional medicinal uses. Apricots, a primary stone fruit produced in temperate regions, stand out among the *Prunus* species for their global cultivation. Apricots are known for a balanced composition of sugars and organic acids and a distinctive aroma. They are predominantly produced in Mediterranean countries. Consuming foods rich in flavonols, such as apricots, has been linked to a lower incidence of chronic diseases. The demand for apricots is on the rise, attributed to their substantial biochemical composition and superoxide scavenging activities. The bioactive compounds in apricots, including polyphenols, contribute to their antioxidative, anti-inflammatory, hepatoprotective, and anti-cancer benefits [14]. The development of a new phytochemical-rich apricot cultivar necessitates an understanding of the phytochemical diversity among various apricot cultivars. The global perspective on daily nutrition is witnessing a transformative shift towards functional foods and natural remedies derived from medicinal plants, driven by the increasing recognition of the therapeutic potential of their bioactive components. This paradigmatic evolution is underscored by the escalating threat of antibiotic resistance and the imperative for alternative therapies. The study of phytochemical diversity among plant cultivars, exemplified by apricots, stands as a crucial endeavor in this context. By analyzing polyphenolic and bioactive compounds in ten apricot cultivars, this research addresses a significant gap in understanding the variability of bioactive compounds within the same species, thereby contributing to the broader discourse on functional foods and natural remedies for disease prevention and treatment. This exploration aligns with the growing interest in leveraging nature-derived remedies for their potential health benefits, including antioxidative, anti-inflammatory, hepatoprotective, anti-cancer, and anti-diabetic properties. Moreover, it underscores the importance of natural antioxidants in mitigating oxidative stress-related diseases, such as cancer, diabetes mellitus, and neurodegenerative disorders. This is in line with previous literature emphasizing the role of bioactive compounds in combating oxidative stress [[1], [2], [3],^5^,^6^,^13^].

## 2 Material and methods

Ten apricot varieties, *viz* Harcot, Hartlay, Rival, Tilton, F. Medester, Chinese, New Castle, Irani, Cummins and Afghani *etc*., were taken at maturity stage during 2020.The maturity stage was determined based on standard horticultural indicators such as color change, fruit firmness and soluble solids content. All apricot varieties were sourced from the Central Institute of Temperate Horticulture (CITH) in Srinagar, India. This institute was selected due to its reputation and expertise in temperate horticulture, ensuring the plants were grown under controlled and standardized conditions. The apricots were cultivated under identical environmental conditions such as similar soil types, irrigation practices and pest management protocols to minimize variability due to external factors.

### 2.1 Sample preparation

To mitigate the oxidation of phenolic compounds, fruits from each variety were homogenized using a mortar and pestle and subsequently quenched in liquid nitrogen at a ratio of 1:2 (w/v) [15]. This process was performed to prepare the material for immediate freeze-drying, excluding the seeds. Homogenization of the freeze-dried fruit material was achieved via further grinding in a mortar. For the extraction process, 8 g of the powdered fruit sample was accurately weighed and transferred into extraction tubes. To each tube, 10 mL of acetone at predetermined concentrations was added. The samples were incubated at 10 °C for duration of 10–15 min to facilitate the extraction of phenolic compounds. Following incubation, the mixtures were subjected to centrifugation using a Sigma 3–30 K centrifuge (Sigma, Munich, Germany) set at 8160×*g* for 20 min at a controlled temperature of 4 °C. The supernatants were then concentrated by vacuum evaporation at 40 °C using an IKA HB-10 rotary evaporator (IKA, Germany) and subsequently lyophilized. The lyophilized extracts were re-dissolved in 3 mL of a solvent mixture composed of 2.5 % acetic acid and methanol in a 3:1 (v/v) ratio. This solution was then filtered through a 0.22 μm nylon syringe filter (Moxcare, Haryana, India) to remove particulate matter, rendering the extracts suitable for subsequent analytical evaluations.

### 2.2 Total saponin content

The methodology used for the determination of total saponin content followed the procedure established by Nguyen [16]. Initially, the samples underwent extraction three times using ethanol, followed by drying using a rotary evaporator at 55 °C. Subsequently, the ethanol-extracted material was dissolved in water and subjected to chloroform extraction to eliminate lipids. A final extraction was then performed using n-butanol. The n-butanol extract was concentrated to a constant mass via rotary evaporation. The total mass of saponins is represented by the dry mass of the n-butanol extract.

### 2.3 Determination of alkaloids

The presence of alkaloids was verified using Dragendorff's method, as reported by Ajanal [17]. A portion of the extract was dissolved in diluted hydrochloric acid, followed by the addition of two drops of Dragendorff's reagent. The crystalline precipitate formed signifies the presence of alkaloids. Samples testing positive for alkaloids were subsequently subjected to quantitative analysis.

### 2.4 Estimation of total phenolic content (TPC)

The determination of total phenolic content was conducted using the method proposed by Slinkard and Singleton [18]. The absorbance of the sample was recorded at 760 nm using a double beam UV–VIS spectrophotometer. The total phenolic content was quantified and expressed in terms of milligrams of gallic acid equivalents (mg GAE) per gram of fresh weight.

### 2.5 Estimation of total flavonoid contents

The flavonol content was assessed using the procedure described by Zhishen [19]. The reaction mixture's total volume was increased to 2.5 mL using distilled water, and its absorbance was determined using a double-beam UV–Visible spectrophotometer at 510 nm. The content of flavonoids was estimated by referring to a catechin standard curve, and the findings were presented in milligrams per gram of fresh weight (mg/g FW)

### 2.6 Estimation of total tannins contents

The quantification of tannin content was performed using a modified methodology derived from the protocol described by Xu and Chang [20]. Absorbance readings were recorded at 500 nm. The amount of tannins was calculated and reported in milligrams of catechin equivalents (mg CE) per gram of fresh weight.

### 2.7 Determination of antioxidant activity

#### 2.7.1 DPPH (2,2-diphenyl-1-picrylhydrazyl) scavenging activity

The approach for evaluating the DPPH radical scavenging activity of the extract was modified from the technique described by Pavic [21]. Absorbance was recorded at 517 nm utilizing a UV/VIS spectrophotometer (Labomed, USA). The scavenging activity of free radicals was quantified in terms of percentage inhibition, employing the following formula:

% inhibition = 100 × (Absorbance of blank - Absorbance of sample) / Absorbance of blank.

#### 2.7.2 FRAP (ferric reducing antioxidant power assay)

The Ferric Reducing Antioxidant Power (FRAP) assay was performed in accordance with the method established by Benzie and Strain [22]. The absorbance of the mixture was determined at 593 nm, using a reagent blank as the reference, after duration of 4 min. The FRAP value was calculated in terms of millimoles of ferrous ion (Fe^2+^) equivalents per gram of fresh weight, utilizing a standard calibration curve derived from ferrous sulfate.

#### 2.7.3 HPLC analysis

The quantification of phenolic compounds in different apricot varieties was performed using a high-performance liquid chromatography (HPLC) system from Shimadzu (Kyoto, Japan), which was equipped with quaternary pumps, a degasser, a photodiode array detector, and a sample injection valve featuring a 20 μL loop. This method, which was modified from the one proposed by Shafi [23], included the detection of catechin and epicatechin at 280 nm, coumaric acid at 345 nm, and rutin at 260 nm. The mobile phase consisted of 2.5 % HPLC-grade glacial acetic acid (Solvent A) and acetonitrile (Solvent B), following a gradient program that started with 3–9% B for the first 0–5 min, escalated to 16–36.4 % B between 15 and 33 min, and finally reached 100 % B for the last 5 min. The analysis was carried out with an injection volume of 20 μL and a flow rate set at 1.0 mL/min, resulting in a total analysis time of 60 min. Each sample was analyzed in triplicate. The quantitative analysis was based on the comparison of the standards' peak areas at specific wavelengths with the concentration, which was reported in micrograms per gram (μg/g) of the apricot sample.

#### 2.7.4 α-amylase inhibitory activity assay

The evaluation of α-amylase inhibitory activity of the extracts was performed by employing a modified method described by Miller [24]. The volume of the reaction mixture was made up to 5 mL using double-distilled water, followed by the measurement of absorbance at 540 nm. A blank solution was created by replacing the enzyme and the inhibitor in the assay with 200 μL of buffer while maintaining all other conditions unchanged. The inhibitory activity was quantified as a percentage of inhibition, using the specified formula for calculation

α-amylase inhibition (%) = (Abs Control – Abs Sample /Abs Control) × 100

Where, Abs = Absorbance.

#### 2.7.5 α-glucosidase inhibitory activity assay

The assessment of α-glucosidase inhibitory activity was conducted using a modified approach based on Dewi [25]. Absorbance readings were taken at 405 nm both before and following the addition of the substrate. To ascertain the inhibitory activity, control was established by substituting the extract with 10 μL of buffer solution, and comparisons were made. The activity was quantified and expressed as a percentage of inhibition, employing the designated formula for calculation.

α-glucosidase inhibition (%) = (Abs Control - Abs Sample / Abs Control) × 100, where Abs represents absorbance

#### 2.7.6 Acetyl cholinesterase inhibition

The enzymatic activity was evaluated in accordance with the procedure described by Ingkaninan and colleagues [26]., with slight modifications. The reaction was observed for duration of 5 min at 405 nm. The enzyme activity was determined by comparing the velocities relative to that of the assay where the buffer was used instead of the inhibitor (extract). The inhibitory activity was examined utilizing the provided formula.

I% = 100 - (A sample/A control) × 100, where A represents absorbance.

### 2.8 Cytotoxic activity

#### 2.8.1 Sample preparation and culturing of cell lines

A concentration of 20 mg/mL was made by dissolving the extract in DMSO to prepare stock solutions. The cancer cell lines employed in this research comprised PC-3 (prostate cancer), A-549 (lung cancer), MCF-7 (breast cancer), HELA (cervical cancer), and HEK (kidney cancer). These cell lines were procured from the National Center for Cell Science in Pune, India, and the National Cancer Institute. Culturing conditions for all cell lines were maintained at 37 °C.

#### 2.8.2 MTT assay

Cell proliferation inhibition was assessed through the MTT assay, as described by Shah [27], with slight modifications. Absorbance was recorded at 590 nm, and the percentage inhibition was estimated by utilizing the specified formula. % inhibition = (A control 590 – A sample 590)/A control 590 × 100.

#### 2.8.3 Statistical Analysis

In this study, comprehensive statistical analyses were employed to discern patterns and relationships among various cultivars. The analyses included correlation analysis, Principal Component Analysis (PCA), and Hierarchical Cluster Analysis (HCA). Each analysis was performed on triplicate data sets to ensure robustness and reproducibility. The results are presented as the mean ± standard deviation (SD). Statistical computations were carried out using the R software framework. Correlation coefficients were determined through Pearson's correlation test to assess the strength and direction of linear relationships between variables. Additionally, IC_50_ values, indicative of the concentration at which 50 % inhibition is observed, were calculated using GraphPad Prism version 5.0.

## 3 Results and discussion

The results of the phytochemical assays are presented in Table 1. The presence or absence of naturally occurring bioactive compounds was determined in this preliminary phytochemical screening of distinct varieties of *Prunus armeniaca* fruit extracts. The presence of phenols, flavonoids, tannins, alkaloids and saponins components in the different fruit extracts with variable strengths was shown by quantitative and qualitative analysis.

**Table 1:** Data represents the variability in the phytochemical composition and antioxidant potential of diverse apricot cultivars.

Cultivar	Phenols (mg GAEs/g FW)	Flavanoids(mg QEs/g FW)	Tanins	Alkaloids	Saponins	DPPH IC_50_ (μg/g FW)	FRAP mM Fe^2+^ eq./g FW
Harcot	33.13 ± 15.21	20.40 ± 10.08	++	+	–	92.03 ± 12.02	1.99 ± 1.08
Hartlay	60.39 ± 11.12	39.49 ± 13.05	+	++	–	61.68 ± 15.04	3.79 ± 1.23
Rival	42.62 ± 16.15	17.40 ± 12.11	++	++	++	81.01 ± 18.22	3.41 ± 2.11
Tilton	106.37 ± 20.05	49.38 ± 11.21	+++	++	+	32.03 ± 20.56	6.76 ± 3.09
F.medester	96.40 ± 11.00	45.22 ± 11.17	++	+++	++	48.21 ± 15.26	5.38 ± 5.21
Chinese	41.52 ± 11.14	26.47 ± 12.18	+	++	+	84.25 ± 12.17	3.68 ± 6.11
New Castle	72.66 ± 17.13	28.42 ± 10.16	++	+	–	46.06 ± 12.12	3.27 ± 7.07
Irani	137.23 ± 18.15	51.26 ± 13.35	+++	++	+++	21.32 ± 11.17	7.62 ± 5.15
Cummins	67.82 ± 14.23	42.63 ± 2.12	+	++	+	51.04 ± 12.21	5.48 ± 8.04
Afghani	55.34 ± 11.00	38.27 ± 16.15	++	+	+	71.27 ± 13.11	4.25 ± 7.14

The data is presented in mean ± SD (n = 3).

### 3.1 Total phenols and flavonoids

The total phenolic content (TPC) of methanolic extracts from ten apricot cultivars was determined and ranged from 33.13 ± 15.21 to 137.23 ± 18.15 mg GAEs/g FW (gallic acid equivalents per gram of fresh weight), as presented in Table 1. Among the assessed cultivars, ‘Irani’ exhibited the highest TPC (137.23 ± 18.15 mg GAEs/g FW), followed by ‘Tilton’ (106.37 ± 20.5 mg GAEs/g FW). In contrast, ‘Harcot’ displayed the lowest TPC (33.13 ± 15.21 mg GAEs/g FW).The total flavonoid content (TFC) of fruit extracts from various apricot varieties was quantified in terms of mg QEs/g FW (milligrams of catechin equivalents per gram of fresh weight of the extract). Substantial variation in TFC was observed among different apricot varieties, with values ranging from (17.40 ± 12.11–51.26 ± 13.35 μg QEs/g FW). The variety Irani depicted the highest TFC (51.26 ± 13.35 μg QEs/g FW), followed by Tilton (49.38 ± 11.21 mg catechineq/g FW). Conversely, the variety Rival exhibited lower TFC content (17.40 ± 12.11 μg QEs/g FW). Our findings align with previous investigations by Sochar [28], Rampáčková [29] and Wani [30] on apricot cultivars. While some bioactive components are common across fruits and vegetables, their concentrations may vary among species or cultivars. Genetic factors play a significant role in determining the content of bioactive compounds in fruits and vegetables. Additionally, factors such as geographical location, cultivation conditions, harvesting time and soil composition can also contribute to variations in phenolic compounds. Prior studies have also noted variability in TPC and TFC content across various fruits, including fresh apricot fruit, almond and blackberry [[31], [32], [33], [34], [35]].

### 3.2 Tannins, alkaloids and saponins

The methanolic fruits extracts were evaluated for their quantitative analysis of tannins, alkaloids and saponins. Each of the fruit extracts showed the presence of tannins and alkaloids, while a majority also tested positive for saponins. The presence or absence of these phytoconstituents in the extracts is summarized in Table 1. Previous studies have also highlighted the presence of tannin content across various species *Prunus*. Tannins, known for their bitter taste, are categorized under phenolic compounds and are recognized for their beneficial health effects, including anti-hypercholesterolemic, anti-hypertensive, and other cardiovascular benefits. Alkaloids are a class of nitrogen-containing organic compounds predominantly found in plants. These compounds are characterized by their pronounced pharmacological effects and are frequently utilized for their medicinal properties. Alkaloids possess potential anticancer properties due to their ability to disrupt microtubules by binding to beta-tubulin, thereby hindering the formation of the mitotic spindle fiber crucial for cell division [36]. Saponins are glycosides possessing a distinctive foaming property. These compounds exhibit a wide range of therapeutic potentials, including antiviral, anticancer and anti-inflammatory effects, contributing to their significance in various fields, including medicine and nutrition [37]. Studies have shown that plant-derived saponin compounds also possess antibacterial, antioxidant and immune-enhancing properties [38]. Comparative transcriptomic analysis and differential gene expression studies suggest that leaf and fruit tissues are primary sites for saponin biosynthesis [39]. Screening plants for phytochemicals is essential for identifying potential novel compounds for medicinal use, as secondary metabolites from plants form the active components of many pharmaceuticals [40]. The variety of secondary metabolites, including alkaloids, glycosides, and tannins found in plants, have significant therapeutic properties and often contribute to their medicinal value [41].

### 3.3 Antioxidant potentials

#### 3.3.1 Free radical scavenging (DPPH)

The antiradical potential of various apricot varieties was evaluated based on their potential to neutralize DPPH free radicals. Table 1 presents the results of the DPPH assay, including the IC_50_ values, which denote the concentration of extract needed to achieve a 50 % reduction in DPPH radical activity, expressed in μg/g of fresh weight (FW). The IC_50_ values for the apricot fruit extracts ranged from 21.32 ± 11.17 to 92.03 ± 12.02 μg/gFW. The Irani variety depicted the strongest radical scavenging ability with an IC_50_ of 21.32 ± 11.17 μg/gFW, followed by the Tilton variety at 32.03 ± 20.56 μg/gFW. Conversely, the Harcot variety exhibited the weakest activity, with an IC_50_ of 92.03 ± 12.02 μg/gFW. These findings align with prior research by Sochor [28], Wani [30] and Olimpia [42], who investigated the antioxidant capacity across various *Prunus* varieties. Similar variability in antioxidant potential among cultivars has been previously documented, suggesting influences of genetic differences, environmental conditions and maturity stages on antioxidant capacity [43,44]. The antioxidant properties of the fruit extracts may be attributed to their polyphenolic content, which is known for its effective radical scavenging actions [[45], [46], [47]]. Methanolic extracts, in particular, may exhibit higher antioxidant activities due to the presence of flavonoids and their ability to donate hydrogen atoms. Previous research has indicated that medicinal plants rich in polyphenolic compounds tend to exhibit pronounced antioxidant properties [[48], [49], [50], [51]]. Moreover, the presence of secondary metabolites such as tannins, glycosides, and alkaloids in the extracts might augment their capacity to combat oxygen radicals.

#### 3.3.2 FRAP

The antioxidant potential of various apricot cultivars was also assessed through the ferric-reducing antioxidant power (FRAP) assay, and the results are summarized in Table 1. In this assay, ferric ions undergo reduction to the ferrous form in the presence of an antioxidant, resulting in the formation of a blue-colored ferrous tripyridyltriazine complex (Fe^2+^+-TPTZ) at pH 3.6. The change in color was spectrophotometrically measured at 593 nm, with results expressed in mMFe^2+^eq./g FW of extract. The FRAP activity of the extracts varied from 1.99 ± 1.08 to 7.62 ± 5.15 mMFe^2+^eq./g FW, as indicated in Table 1. The variety Irani exhibited the highest FRAP value (7.62 ± 5.15 mMFe^2+^eq./g FW), followed by Tilton (6.76 ± 3.09 mMFe^2+^eq./g FW), while the lowest FRAP value was recorded in Harcot (1.99 ± 1.08 mMFe^2+^eq./g FW). The ferric ion-reducing activities of all fruit extracts displayed a similar trend to that observed in the DPPH assays. Our study's findings concerning Fe^3+^ reducing potential were comparatively higher than those reported by Sochar [28] for Czech Republic apricot fruit and the analysis of Turkish apricot cultivars by Capanoglu [52]. The FRAP assay is recognized for its high reproducibility and rapid execution [53]. The observed reducing properties are often ascribed to the extracts' hydrogen-donating potential, enabling them to disrupt the free radical chain [54]. The notable variation in free radical scavenging potential among different fruit varieties in the FRAP assay may be attributed to discrepancies in their chemical compositions. The FRAP assay signifies that the tested samples possess the capability to donate electrons to free radicals in various food and biological processes [55]. The outcomes of the two antioxidant methods for extracts from the ten different apricot cultivars in this study were concurrent; each test demonstrated distinct antioxidant activity, highlighting the influence of both sample composition and procedural conditions on antiradical activity [56].

### 3.4 HPLC analysis

Based on the fact that antioxidants are closely related to polyphenolic content, quantification of five (5) polyphenolics was carried out in ten (10) apricot cultivars (Table 2). The maximum catechin content was observed in variety Irani (241.00 ± 26.12 μg/g FW), and the minimum catechin content (27.00 ± 14.25 μg/g FW) was observed in variety F. medester. The maximum epicatechin content was observed in the apricot cultivar Irani (504.00 ± 16.55 μg/g FW), and the minimum epicatechin content was observed in cultivar Hartlay (28.00 ± 18.55 μg/g FW). Quercetin content was recorded maximum in variety Cummins (228.00 ± 17.10 μg/g FW), followed by Chinese apricot (171.00 ± 15.42 μg/g FW), and the minimum Quercetin content was observed in New Castle (3.00 ± 1.55 μg/g FW). The maximum coumaric acid content was observed in the cultivar Irani (897.00 ± 28.65 μg/g FW), and the minimum coumaric acid content was observed in Chinese apricot (16.00 ± 11.82 μg/g FW). Rutin was found highest in variety Cummins (75.00 ± 12.29 μg/g FW), which was followed by a variety Irani (46.00 ± 11.21 μg/g FW). The minimum Rutin content was recorded in a variety Chinese Apricot (11.00 ± 3.09 μg/g FW). HPLC study offers complete quantitative and qualitative information about the polyphenolic compounds present in the extracts than TPC estimated by the Folin-Ciocalteu method. Among the five standard phenolic compounds used in this study for their presence in the methanolic fruit extracts of different apricot varieties, coumaric acid was found in higher amounts in the variety Irani. The qualitative and quantitative composition of phenolics in fruits is conventional and exclusive for individual species and genotypes [47,57] and can be utilized for separating their chemotaxonomy. In our analysis, a significant variation of polyphenolic content recorded has also been reported in a previous study [30]. Polyphenolic content also depends on the type of cultivar and their genetic makeup [58,59]. These polyphenols quantified in different apricot varieties in this analysis may be responsible for the health-related benefits, as prior reports have already described the pharmacological properties of these flavonols [60].

**Table 2:** Data represents the variability of different bioactive molecules in different apricot cultivars.

Cultivar	Catechin (ug/gFW)	Epicatechin (ug/gFW)	Quercetin (ug/gFW)	Coumaric acid (ug/gFW)	Rutin (ug/gFW)
Harcot	91.00 ± 33.25	52.00 ± 14.25	65.00 ± 31.55	126.00 ± 44.68	25.00 ± 14.62
Hartlay	66.00 ± 45.25	28.00 ± 18.55	22.00 ± 17.59	141.00 ± 40.92	38.00 ± 13.43
Rival	46.00 ± 53.25	75.00 ± 15.58	Nd	127.00 ± 28.17	16.00 ± 11.87
Tilton	36.00 ± 33.58	194.00 ± 21.11	126.00 ± 23.51	257.00 ± 55.74	42.00 ± 19.27
F.medester	27.00 ± 14.25	Nd	21.00 ± 34.80	153.00 ± 27.67	30.00 ± 17.19
Chinese Apricot	123.00 ± 22.15	55.00 ± 23.32	171.00 ± 15.42	16.00 ± 11.82	11.00 ± 3.09
NewCastle	Nd	67.00 ± 13.83	3.00 ± 1.55	214.00 ± 27.97	12.00 ± 9.29
Irani	241.00 ± 26.12	504.00 ± 16.55	158.00 ± 12.25	897.00 ± 28.65	46.00 ± 11.21
Cummins	62.00 ± 56.93	64.00 ± 37.59	228.00 ± 17.10	115.00 ± 26.33	75.00 ± 12.29
Afghani	214.00 ± 76.01	56.00 ± 10.21	42.00 ± 17.45	96.00 ± 24.47	28.00 ± 12.31

The data is represented in mean SD± (n = 3).

#### 3.4.1 α-amylase and α-glucosidase inhibitory activity

Diabetes results in extreme complications, which can be specified by elevated sugar levels in the blood. To prevent the diabetic effects in the body, maintaining glucose levels is crucial. Currently, there is no cure or drug available to treat diabetes without adverse effects [61]. Medications that obstruct the degradation of disaccharides to monosaccharides are commonly referred to as oral hypoglycemic agents because they prevent this conversion, thus maintaining blood sugar levels [62]. Pancreatic α-amylase, one of the main enzymes in the digestive system, is involved in the degradation of starch into disaccharides and oligosaccharides, thereby liberating glucose for absorption into the bloodstream. Inhibition of amylase can reduce starch digestion in the gastrointestinal tract, consequently decreasing the degree of postprandial hyperglycemia. The capacity of different cultivars to inhibit α-amylase and α-glucosidase was investigated. Although all the varieties tested showed good percentage inhibition of the enzymes, however there were notable variances in their efficiency. The range of inhibition values was recorded between 46.97 % and 88.71 %, respectively. These values for different varieties are presented in Fig. 1a. The percentage inhibition in our analysis was comparable to the study on fruit extracts of *Passiflora ligularis* and different fractions of the labiatae plant, and higher than the study carried out by Kifle [63]. Plant extracts with higher polyphenols content tend to have a greater potential to suppress the α-amylase enzyme [64]. Therefore, the high polyphenols content in extracts of *P. armeniaca* fruit may be the reason for the inhibitory activity. In the current study, α-glucosidase inhibitory percentage was also measured among the different cultivars of apricot. The different cultivars showed a good percentage of inhibitory potential, with the range of inhibition varying from 36.39 % to 83.59 %, as presented in Fig. 1b. The higher percentage of inhibition was shown by variety Irani (83.59 %), while the lowest inhibition potential was seen in variety Harcot (36.39 %). Polyphenolic components derived from plants have traditionally been considered to alter glucose consumption in animals, resulting in insulin and anti-obesity activities [65]. Earlier studies on different fruit extracts, such as raspberry, strawberry, and grape, have also revealed that different flavonols are responsible for inhibiting α-amylase and α-glucosidase [66].

**Fig. 1:** Graphs represent the inhibitory potential of different Prunus armeniaca fruit extracts at a concentration of 100 μg/mL. Values are the mean ± SD (n = 3).

Our findings indicate that apricot cultivars possess significant inhibitory activity against α-amylase and α-glucosidase, suggesting their potential role in managing postprandial hyperglycemia. The variation in inhibition percentages among different cultivars underscores the influence of specific phytochemical compositions, particularly polyphenols, which have been shown to enhance the inhibitory effects on these digestive enzymes [64]. This aligns with the results observed in other fruit extracts, where high polyphenolic content correlates with increased enzyme inhibition [66]. The potent inhibitory activity of the Irani cultivar, as demonstrated by its high percentage of inhibition against α-glucosidase, highlights the potential of certain apricot varieties to be utilized as natural sources for developing oral hypoglycemic agents. Moreover, the inhibition of α-amylase and α-glucosidase is a well-recognized strategy for controlling diabetes, as these enzymes play critical roles in the breakdown of carbohydrates, thereby influencing blood glucose levels [67]. Plant-derived polyphenolic compounds, such as flavonoids, tannins, and phenolic acids, have been extensively studied for their ability to inhibit these enzymes and mitigate hyperglycemia [68]. For example, the flavonols present in raspberry, strawberry and grape have been shown to effectively inhibit these enzymes, contributing to their anti-diabetic properties [66]. Furthermore, the potential anti-diabetic effects of polyphenols extend beyond enzyme inhibition. They have been reported to enhance insulin sensitivity, reduce inflammation, and exert antioxidant effects, which collectively contribute to their therapeutic benefits in diabetes management [69]. The high polyphenolic content in apricot cultivars not only supports their enzyme inhibitory activity but also suggests additional health benefits that could be advantageous in managing diabetes and its complications [70]. Therefore, the integration of apricot extracts, particularly those from high-inhibition cultivars like Irani, into dietary regimens or as complementary therapies could offer a natural and effective approach to diabetes management. Further research is warranted to isolate and characterize the specific polyphenolic compounds responsible for these effects and to evaluate their clinical efficacy and safety in diabetic patients [71].

#### 3.4.2 Acetylcholinesterase inhibitory activity

Alzheimer's disease (AD) is an age-associated neurodegenerative disorder characterized by progressive memory impairment that ultimately culminates in dementia. Current therapeutic strategies predominantly focus on ameliorating symptoms by modulating neurotransmitter levels, particularly through the inhibition of acetylcholinesterase (AChE). This enzyme degrades the neurotransmitter acetylcholine (ACh), and its inhibition is crucial for maintaining adequate neurotransmitter levels at synaptic junctions, thereby potentially alleviating cognitive decline observed in AD patients [72].The discovery of natural compounds with AChE inhibitory activity is of significant interest. Plant-derived bioactive compounds offer a promising reservoir for novel AChE inhibitors, providing a foundation for the development of new therapeutic agents against neurodegenerative disorders such as Alzheimer's disease. Hence, research into phytochemicals that inhibit acetylcholinesterase is essential for advancing our understanding of their mechanisms and potential efficacy in the treatment of Alzheimer's disease and related neurological conditions. The inhibitory potential of different apricot cultivars against AChE was assessed, and the results are presented in Fig. 1c. The inhibitory potential against AChE varied considerably among the studied apricot extracts. The range of values for different varieties was observed between 53.91 % and 87.13 %, as depicted in Fig. 1c. The inhibitory capacity of the extracts against AChE was comparable to that measured by Paulina [73] in peach kernels. Additionally, the outcomes of our findings were similar to the study conducted by Zengin [74] on medicinal plants such as *Hedysarumvarium*, *Onobrychishypargyrea*, and *Viciatruncatula*. Earlier investigations have also revealed that ayurvedic medicinal herbs have greater potential to inhibit AChE. Reactive oxygen species are known to play a significant role in cell deterioration and are among the initial events in Alzheimer's disease [75]. Therefore, plants containing natural bioactive compounds such as flavonoids, which exhibit antioxidant properties and other promising effects, could be recognized as favorable agents in combating and treating Alzheimer's disease. Numerous studies have reported that medicinal plant products can prevent diseases caused by oxidative stress by slowing the oxidation of lipids or other molecules and preventing the spread of oxidative chain reactions [76]. Some studies have discovered that a group of flavonoids tends to suppress the activity of pro inflammatory cytokines, leading to a reduction in the synthesis of TNF-α and IL-1β produced in microglia, which are responsible for the effects of Alzheimer's disease [77]. Therefore, apricot can be a valuable source of polyphenols to aid in managing Alzheimer's disease.

#### 3.4.3 Anti-cancer activity

The cytotoxic activity of methanolic fruit extracts from differentapricot varieties was evaluated against a panel of human cancer cell lines, including cervical (HELA), kidney (HEK), breast (MCF-7), prostate (PC-3), and lung (A-593) using the MTT assay. The results demonstrated varying percentage of cytotoxicity across all five human cancer cell lines at a concentration of 20 mg/mL. Different methanolic fruit extracts exhibited distinct levels of inhibitory percentages, as presented in Fig. 2. Among all the 10 extracts, Irani and Tilton showed significant inhibitory effects across all cell lines, particularly in the breast cancer cell line MCF-7. Cultivar Irani exhibited growth inhibition ranging from 51 % to 89 %, while Cultivar Tilton showed inhibition percentages between 19 % and 84 %, respectively. Methanolic extract of *Prunus armeniaca* kernel has been screened earlier also for its in vitro anticancer activity against various human cancer cell lines and has shown potential against breast, bladder, lung and liver cancers [78]. In 2018, the incidence of cancer increased to 18.1 million new cases and 9.6 million fatalities. Men primarily experience colorectal, liver, lung, prostate, and stomach cancers, while women are more susceptible to breast, cervical, colorectal, lung, and thyroid cancers [79]. Amygdalin, a major compound in *Prunus armeniaca*, has been found to reduce the viability of SK-BR-3 cells and induce apoptosis through modulation of Bcl-2 and Bax protein expression [80]. Previous studies have reported the cytotoxic effects of amygdalin in various cancer cells, including, lung cancer, prostate cancer, bladder cancer, renal cell carcinoma, triple-negative breast cancer and human cervical cancer [[81], [82], [83], [84], [85]].

**Fig. 2:** Graphs represent *invitro* cytotoxic potential of different cultivars of *Prunus armeniaca* fruit extracts at concentration 20 μg/mL. Values are the mean ± SD (n = 3).

The study of cancer treatment has expanded significantly, with various approaches such as chemotherapy, radiation therapy and surgery, as well as traditional and contemporary methods. However, each of these methods has drawbacks [86]. Natural compounds have long been of interest in cancer treatment due to their therapeutic properties. Plants derived products have been widely studied to identify novel chemicals for cancer treatment [87]. Apricots have been extensively studied for their pharmacological effects, including antiparasitic, anti-cancer, anti-ageing, antiatherosclerosis, antianginal and antioxidant properties, among others [[88], [89], [90], [91], [92], [93], [94]]. Our findings indicate that different apricot fruit extracts exhibited significant in vitro cytotoxicity against the breast cancer cell line MCF-7 compared to other cell lines. Variations in the response of cancer cells to the same cytotoxic agent may be attributed to differences in genetic makeup, morphology and doubling time, leading to variable resistance [95]. Previous reports have also demonstrated strong in vitro cytotoxic effects of apricot fruit on breast cancer cell lines. Compounds extracted from *prunus* species have been found to downregulate NFκB and PD-L1 expression and enhance T cell cytotoxicity against cancer cells [96,97]. The natural combination of cytotoxic agents can impact cell cycle progression, suppress cellular growth, and induce tumor cell death via apoptosis or autophagy. Our findings corroborate the significant cytotoxic potential of methanolic apricot fruit extracts against various human cancer cell lines, particularly the breast cancer cell line MCF-7. The pronounced inhibitory effects of Cultivars Irani and Tilton highlight the potential of these extracts as promising candidates for further exploration in cancer treatment. The observed variability in cytotoxicity across different cancer cell lines underscores the complex interplay between phytochemicals and cancer cell biology [95]. This variability is crucial in understanding the selective cytotoxicity of natural products and tailoring more effective and targeted cancer therapies. Moreover, recent research has emphasized the role of bioactive compounds in inducing apoptosis and autophagy in cancer cells, contributing to their anti-cancer properties [98]. Additionally, apricot extracts have shown potential in downregulating pro-survival pathways and promoting cell death mechanisms, which are crucial for effective cancer treatment [99,100].The therapeutic promise of apricot-derived compounds extends beyond their cytotoxic effects. They also exhibit anti-inflammatory and antioxidant properties, which can contribute to their overall anti-cancer efficacy by reducing oxidative stress and inflammation in the tumor microenvironment [101,102]. Furthermore, the integration of natural compounds into conventional cancer therapies has been suggested to enhance treatment outcomes while minimizing adverse effects [103]. Therefore, continued research into the bioactive constituents of apricot extracts and their mechanisms of action is essential for advancing our understanding of their therapeutic potential in oncology. By elucidating the molecular interactions and pathways affected by these natural compounds, we can develop more effective and less toxic cancer treatments, potentially improving patient outcomes and quality of life [104,105].

#### 3.4.4 Statistical Analysis

The correlation analysis conducted in this study revealed that phenols are highly correlated with flavonoids (r = 0.92), DPPH (r = 0.95) and alpha-amylase (%) inhibition (r = 0.96) and exhibited a significant correlation with other parameters. Similarly, it was observed that flavonoids were highly correlated with DPPH, FRAP and alpha-amylase (%) inhibition and significantly correlated with other parameters. The correlation between flavonoids and antioxidant activity may explain the antioxidant activity of apricot cultivars [106], which suggested that the antioxidant activities of apricot cultivars could be largely attributed to their flavonoid content. Additionally, prior studies have established a significant relationship between polyphenols and antioxidant capacities, suggesting that polyphenols play a critical role in inhibiting oxidative chain reactions within biological systems. Moreover, the positive correlations observed between TPC, TFC, and **Statistical Analysis**.

#### 3.4.5 Statistical Analysis

The correlation analysis conducted in this study as depicted in Fig. 3, revealed that phenols are highly correlated with flavonoids (r = 0.95), DPPH (r = 0.91) and alpha-amylase (%) inhibition (r = 0.94) and exhibited a significant correlation with other parameters. Similarly, it was observed that flavonoids were highly correlated with DPPH, FRAP and alpha-amylase (%) inhibition and significantly correlated with other parameters. The correlation between flavonoids and antioxidant activity may explain the antioxidant activity of apricot cultivars [106], which suggested that the antioxidant activities of apricot cultivars could be largely attributed to their flavonoid content. Additionally, prior studies have established a significant relationship between polyphenols and antioxidant capacities, suggesting that polyphenols play a critical role in inhibiting oxidative chain reactions within biological systems. Moreover, the positive correlations observed between TPC, TFC, and the inhibition of alpha-amylase and alpha-glucosidase align with recent research, including studies by Shan [107] and Rosman [108]. These studies have demonstrated that TPC and TFC are closely associated with the inhibition of digestive enzymes, underscoring the potential of these compounds as natural inhibitors. This evidence collectively suggests that the phenolic and flavonoid profiles of apricot cultivars significantly contribute to their antidiabetic and antioxidant potential, offering a valuable basis for further exploration of their therapeutic potentials.

**Fig. 3:** Correlation Plot of different parameters.

The upper triangular matrix presents Pearson correlation coefficients along with significance levels indicated by stars. Each significance level is represented by a symbol: p-values 0.001 are marked as (∗∗∗), 0.01 as (∗∗) and 0.05 (∗).This plot was created using R programming language.

**Principal Component Analysis**. PCA was conducted simultaneously on all variables to identify the pattern of variation using R Studio (R-4.2.1). Principal axis 1 (PC1) accounted for 43.31 % of the variance, while principal axis 2 (PC2) accounted for 12.88 %, together explaining 80.033 % of the total variance of the data matrix, with PC1 being the dominant axis. Factor loading, ranging from −1 to 1, measures the correlation between the original variables and the factors created via PCA. A value of −1 or 1 indicates a significant association, while a value close to 0 indicates a weak correlation.

Fig. 4 illustrates the classification based on factor scores. The variable biplot effectively reveals the visual comparison of all fractions based on multiple parameters, demonstrating the relationships between variables. Important data were obtained using the angles formed by the vectors and the distance of the fractions from the biplot's origin. When the angle between two variable vectors is less than 90°, there is a positive correlation, while an angle greater than 90° indicates a negative correlation. A 90-degree angle indicates no correlation between the parameters [109]. In the biplot, the angle between DPPH and HELA can be observed as equal to 90°, indicating no correlation between these two parameters.

**Fig. 4:** Loading plot of variable parameters.

In Fig. 5, the scree plot presents eigen values in a descending curve, arranged from the largest to the smallest. The plot identifies the elbow, where the eigen values start to stabilize, indicating significant factors or components to retain on the left side of this point. The scree plot visualizes the amount of retained data. In PCA1, 43 % of the data explains the variation, while PCA2 justifies 12 % of the variation. The variability observed in PCA3, PCA4, PCA5, PCA6, PCA7, PCA8, PCA9, and PCA10 is 8.7 %, 8.4 %, 6.4 %, 6.2 %, 5.5 %, 4.5 %, 4.1 %, and 0 %, respectively. More data is concentrated in PCA1, indicating superior performance compared to the other values. A higher percentage of retained data corresponds to better data performance.

**Fig. 5:** Scree plot showing eigen value and cumulative variability of studied parameters.

To assess the similarity among the cultivars, Hierarchical Cluster Analysis (HCA) was conducted (see Fig. 6). The HCA resulted in the division of cultivars into 2 main clusters, with cluster 2 further subdivided into various sub-clusters and sub-sub-clusters. Cluster 1 comprised only 1 cultivar, Irani. According to the cluster analysis, all cultivars except Irani were grouped in cluster 2, indicating a close genetic resemblance among them. The separation of Cultivar Irani into a distinct cluster may be attributed to its different genetic nature, suggesting less similarity with other cultivars [110]. This differentiation could account for its higher antioxidant potential and prominence in polyphenolic compounds compared to other cultivars.

**Fig. 6:** Schematic representation displaying the clustering pattern of 10 different apricot cultivars.

## 4 Conclusion

The present investigation underscores the substantial impact of variability on phytochemical composition and health-promoting attributes among distinct apricot cultivars. Notably, this study unveils, for the first time, the potent anti-cancer efficacy of two specific apricot varieties, namely Irani and Tilton, particularly against the MCF-7 breast cancer cell line. These cultivars manifest the highest levels of bioactive constituents among the evaluated varieties and demonstrate significant inhibition of diabetic enzymes and acetylcholinesterase. Plant-derived bioactive compounds, including alkaloids, saponins, and tannins, exhibit diverse mechanisms in combating serious diseases and ameliorating adverse conditions. Despite promising outcomes from both in vitro and in vivo investigations, thorough evaluation of the bioactivity of individual compounds and their synergistic interactions remains imperative. Subsequent exploration of these bioactive compounds, elucidating their distinct roles in disease management, is crucial for their potential commercialization as pharmaceutical alternatives or dietary supplements, thereby advancing healthcare paradigms. While in vitro assays provide valuable insights into the potential therapeutic effects of apricot extracts but they do not fully represent the complex interactions that occur in vivo. Consequently, future endeavors should integrate animal models to validate the observed anti-cancer and anti-diabetic effects. Furthermore, Investigating the underlying molecular mechanisms of action through transcriptomic, proteomic and metabolomic analyses would provide a deeper understanding of how apricot-derived bioactive compounds exert their therapeutic effects.

## Data availability statement

The data presented in this study are available on request from the corresponding author.

## CRediT authorship contribution statement

**Zahid Nabi Sheikh:** Writing – original draft, Validation, Supervision, Methodology, Investigation, Funding acquisition, Formal analysis, Data curation, Conceptualization. **Vikas Sharma:** Writing – original draft, Visualization, Validation, Project administration, Methodology, Investigation, Formal analysis, Data curation, Conceptualization. **Shilpa Raina:** Writing – original draft, Visualization, Software, Resources, Funding acquisition, Formal analysis, Data curation. **Prashant Bakshi:** Writing – original draft, Visualization, Validation, Methodology, Investigation, Formal analysis, Data curation, Conceptualization. **Rizwan yousuf:** Writing – review & editing, Visualization, Validation, Project administration, Methodology, Investigation, Formal analysis, Data curation. **Ali Zari:** Writing – original draft, Supervision, Software, Resources, Project administration, Formal analysis, Conceptualization. **Talal A. Zari:** Writing – original draft, Visualization, Software, Project administration, Methodology, Funding acquisition, Formal analysis. **Khalid Rehman Hakeem:** Writing – review & editing, Writing – original draft, Validation, Project administration, Methodology, Investigation, Funding acquisition, Formal analysis, Conceptualization.

## Declaration of competing interest

The authors declare that they have no known competing financial interests or personal relationships that could have appeared to influence the work reported in this paper.
